The article "Research on Intelligent Scheduling Scheme of Aerobics Competition for Multi-Intelligent Decision-Making" was published in 2022. Journal: Comput Intell Neurosci.

# Research on Intelligent Scheduling Scheme of Aerobics Competition for Multi-Intelligent Decision-Making

**DOI:** 10.1155/2022/3407494

**Published:** 2022-05-23

**Authors:** Hongjing Guan, Zhi Tan, Xingrui Zhao

**Affiliations:** ^1^Graduate School, José Rizal University, Manila 0900, Philippines; ^2^Graduate School, Woosuk University, Jeonju 514500, Republic of Korea

## Abstract

Multi-intelligent decision-making has a good development at present. Based on a series of technologies such as artificial intelligence, multi-intelligent decision-making is involved in many aspects, and the country also attaches great importance to the development of such science and technology. At the same time, at present, the development of the sports industry is not balanced. Even if the country values the sports industry, it needs investment in science and technology. This paper studies the scheduling scheme of aerobics competition in sports competition. By introducing the design scheme of a multi-intelligent decision-making system and improving the MFDRL-CTDE algorithm, the similarity between the action sequence of participants in aerobics competition and the standard action sequence is obtained. Three algorithms including Markov, MFDRL-CTDE algorithm, and improved MFDRL-CTDE algorithm are used for simulation experiments, and the improved MFDRL-CTDE algorithm is more effective and stable for the decision-making of aerobics competition.

## 1. Introduction

Our country is very interested in the development of science and technology. The application of intelligent decision-making system has penetrated into all walks of life, and the application of intelligent decision-making system has also been internationally recognized. Researchers have developed related intelligent decision-making in depth, which greatly improves the performance of various related decision-making algorithms and makes related applications more efficient. While taking care of the development of science and technology, the country pays more attention to the development of sports, especially the development of aerobics competition. The development history of aerobics is not long ago, but it is loved by the broad masses of people, and it has the performance of sports competition while having an aesthetic feeling. However, the development is not balanced, so it is necessary to put science and technology into aerobics competition and intelligent decision-making into aerobics competition, so as to make aerobics competition have better development.

In the process of studying intelligent decision support system, many new methods have emerged [1]. According to the structural characteristics and system characteristics of the system, an improved model can be designed well. Group is the foundation of the organization of individual intelligence, and the model and strategy discussed are also based on this characteristic. Combined with the combination mechanism, the model can run efficiently. The decision-making process plays an important role in the interactive trend of multi-intelligence combination [2]. In order to accurately predict, it is impossible to use probability or theory alone. What game can bring is very good decision-making and identification. The Bayesian game model is the combination of game and graph, which can solve the complex situation caused by multi-intelligent agent interaction. Compared with other intelligent decision information systems, this model has better decision efficiency. Because decision-making and evaluation are not carried out at the same time, their operation process is affected by many factors. Nevertheless [3], it is extremely urgent to improve the efficiency of group decision-making. Therefore, the rational political model is put forward, and its purpose is to improve the operational efficiency of group decision-making in the face of uncertain factors. In this process, this model clarifies the factors. Moreover, this model obtains the best scheme of group decision-making on the basis of a sequence framework when there are different complete evaluations, information, and opinions. In real-time work [4], such as the intensive care unit, what doctors need is the result of matching time and information, and the important value of an intelligent decision support system is the agent of two or more people to complete tasks cooperatively. At present, the architecture of a multiagent system has been proposed, which is undoubtedly to support the decision-making of clinical data and predictive status required by doctors. The artificial neural network algorithm is divided into two steps [5]. The first step is to use the improved algorithm to calculate the relevant weight matrix. The second step is to apply the method to real system decision-making, such as a multi-intelligent robot soccer system. The final simulation results show that this technology can be efficiently used in small- and medium-sized league system decision-making. Multicriteria decision-making method can be applied to aerospace systems effectively [6] and help decision makers to solve related conflict problems. In the face of a variety of multicriteria decision-making methods, we need to choose the appropriate method, but this is a very complex problem related to multicriteria decision-making. The proposal of 14 criteria can evaluate the feasibility of the multicriteria decision-making method, so that the preference of decision makers can be better informationized. If we want to develop an intelligent knowledge system, we can optimize the suitability index. In order to prove the effectiveness of the system, the aircraft selection problem can solve this problem well. In order to realize the UniComBOS of intelligent decision support system [7], we propose to use verbal decision to analyze the paradigm. In this range, for multistandard alternatives, the processing ability of individual decision makers is considered, and the information of decision makers' psychological preferences is accurately extracted on this premise. In the user interface, the decision-maker's psychological preference is distinguished in the form of graphic color, which provides a psychological comparison for the decision-maker and can test whether the decision-maker's answer is consistent. Like conventional decision-making tools, this scheme decomposes the whole part with the least number of criteria, so that the comparison range of decision makers can be reduced to a single criterion, and then, the criteria are added until the advantages of the optimal substitute are found. However, in the case of multiple standards, a single optimal alternative cannot be found by the system, so only a group of alternatives can be found. However, there is no comparability between these alternatives, but they still have great advantages over those that are not selected. In the EFQM excellence model, literature [8] is used to achieve business excellence, which is mostly used for the self-business evaluation of many nonlarge enterprises in Britain. In fact, this is a problem related to multistandard decision analysis. At present, experiments have proved that in order to realize the method of achieving excellent business through action, an intelligent decision system is used to support program groups, which not only makes the average score come out but also can wait for numerical results and graphic comparison. At present, the society is interested in sports as well as the development of science and technology [9]. In Korea, aerobic exercise is popular with people. However, it has been emphasized recently that sports need technology and competition, which makes the development trend of aerobic exercise that shows an unbalanced trend. Among them, the development of aerobics is relatively rapid. In order to find a new way out for aerobics, it is very important to understand its history and introduction process. The demand and rapid change of society for aerobics is the key to the development of aerobics, and the development needs to be carried out in a moderate way and cannot be too radical in any field. According to the data shown, the relevant results of aerobics competition need to be analyzed with various related techniques [10], which can well analyze whether the scores given by the referee are reasonable and consistent. It makes the selection and scoring of referees more scientific and effective. Referees need to maintain an objective and fair attitude towards competition scoring, and rational evaluation can better develop and build the future of aerobics competition. Aerobics Championship needs to analyze the movements [11]. According to the rules, difficulties, and characteristics of the world aerobics competition, each group performs differently. There are outstanding performances in dynamic strength or outstanding performances in balance flexibility, and the most outstanding ones in each group are different. For the analysis of aerobics competition results, we can use related research methods, such as comprehensive omission research and variance analysis [12]. Through the experimental data, we can observe that the scores given by the judges are relatively the same, and of course, the performance displayed by the finished judges is better than that of the artistic judges. Therefore, no matter what kind of aerobics competition, it needs a systematic scoring test program. Relevant technologies are used to simplify scores and evaluate objectively. At the same time, participating members can question scores and arbitrate. According to the statistical analysis of the skills of the first six participants in a certain aerobics competition [13], and summarizing the techniques of music rhythm and aerobic exercise, we can develop ladder aerobics and find out its characteristics. The most important point is that this can make junior coaches have more references for aerobics competition. For students' aerobics competition, on-site observation, interview, and video analysis of the later competition are also very important [14]. This is a strengthening of aerobics education for students and a reference for the competition itself. Our country attaches great importance to the development of gymnastics and aerobics [15], and many related training competitions are held by national-level organizations. However, the future development of aerobics needs to be analyzed through data literature, refers to recent training, and changes to solve the problems on the road of development.

The article "Research on Intelligent Scheduling Scheme of Aerobics Competition for Multi-Intelligent Decision-Making" was published in 2022. Journal: Comput Intell Neurosci.

## 2. Multi-Intelligent Decision Analysis

### 2.1. Basic Concepts

Multi-intelligent decision-making refers to the collective integration of multiple intelligent units, so a huge system is composed of multiagents. One of the main tasks of multi-intelligent decision-making is that decision makers disassemble comparatively complex systems, which is a decision-making process. A complex system is divided into several small systems, and these small systems will be combined again. It should be noted that these small systems are interactive, which is why we can ensure that each system is interactive, so as to improve work efficiency. Compared with other technologies, multi-intelligent decision-making has absolute advantages, which are manifested in its independence, relevance, and application development. The classification of intelligent decision is shown in Figure 1.

### 2.2. Markov

The sequential decision means that after the *t*-th iteration, the state *s* of the environment will be received by the agent, and on this basis, an action *a* will occur. Because the agent and the environment are related to each other, this means that the previous actions will also affect the environment, which will make the agent get a reward, that is, a reward *R*_*t*+1_, so as to stimulate its new state. It is precisely because of the interaction between agent and environment that sequences can be generated. Markov's decision process is to formulate the above process, and Markov's definition formula is as follows:

(1) $$\begin{array}{c} P\left[S_{t+1}|S_{t}\right]=P\left[S_{t+1}|S_{1},\ldots ,S_{t}\right]. \end{array}$$

That is, in Markov, the state of the *t* +  1 iteration and the state of the *t* iteration are related.

State *s* and the state transition probability *p* based on its next state *s*′ are expressed as follows:

(2) $$\begin{array}{c} P_{ss^{\prime }}=P\left[S_{t+1}=s^{\prime }|S_{t}=s\right]. \end{array}$$

That is, in Markov, the state of the *t* + 1 iteration is only related to the state of the *t* iteration.

The formula for getting the reward expectation when the state *s* moves to the next state *s*′ based on it is as follows:

(3) $$\begin{array}{c} R_{s}=E\left[\frac{R_{t+1}}{S_{t}=s}\right]. \end{array}$$

The formula for all rewards and *G* from state *s* to the final state point is as follows:

(4) $$\begin{array}{c} G_{t}=R_{t+1}+\gamma R_{t+2}+\cdots =\sum_{k=0}^{\infty }\gamma^{k}R_{t}+k+1, \end{array}$$

where *γ* is a discount factor, which is a parameter used to express attenuation.

### 2.3. MFDRL-CTDE Algorithm

#### 2.3.1. Multiagent Fuzzy Deep Reinforcement Learning

The main task of a fuzzy inference system is to fuzzify and defuzzify variables. Its core idea is that when the state is input, variables are continuously fuzzified, and the fuzzification of behavior is due to the prescribed rules, and finally, the behavior should be defuzzified and output. When the output variable is controlled at [0, 1], the input fusion weight *w*_*F*_ of the system is the combination of the cumulative average reward and the sample priority in the iteration period, and its normalization formula is as follows:

(5) $$\begin{array}{c} {\bar{w}}_{F}=\frac{w_{F}}{\sum_{i}^{I}w_{F_{i}}}=\left[{\bar{w}}_{F_{1}},{\bar{w}}_{F_{2}},\ldots ,{\bar{w}}_{F_{i}},\ldots {\bar{w}}_{F_{I}}\right], \end{array}$$

where *I* is the total number of agents.

The article "Research on Intelligent Scheduling Scheme of Aerobics Competition for Multi-Intelligent Decision-Making" was published in 2022. Journal: Comput Intell Neurosci.

However, the network parameters *θ* in the system will not be equal to 0 after many iterations, so the formula for updating the parameters is as follows:

(6) $$\begin{array}{c} \theta_{V\text{ tar}}=\sum_{i}^{I}{\bar{w}}_{F_{i}}\theta_{V\text{ val}}^{i},\\ \theta_{A\text{ tar}}=\sum_{i}^{I}{\bar{w}}_{F_{i}}\theta_{A\text{ val}}^{i},\\ \theta_{\text{tar}}=\sum_{i}^{I}{\bar{w}}_{F_{i}}\theta_{\text{val}}^{i}. \end{array}$$

#### 2.3.2. Centralized Training and Decentralized Execution

Each agent affects the value function that determines each of them, which is indispensable in multi-intelligence deep reinforcement learning. Because of this, Markov's decision process in multi-intelligence system is not working well, and the hidden information is difficult to be fully discovered by the agent, so it is necessary to capture this information during training. Centralized training and decentralized execution make use of this point to help agent improve efficiency and, at the same time, store the available information of agent interaction into the shared experience pool, thus further improving efficiency.

For centralized training, the value functions of agents are related to joint behaviors rather than local ones, and they are trained with extra information. For decentralized execution, agent decision-making only depends on the information that has been mined, rather than all the complete information.

## 3. Optimization Algorithm

### 3.1. Optimize MFDRL-CTDE Algorithm

Because of the low fitting ability of the value function in the initial stage, the MFDRL-CTde algorithm cannot guarantee its high efficiency. Therefore, in order to improve the efficiency of the algorithm and reduce the volatility of the algorithm, it is necessary to add competitive DQN and preferential empirical playback. The algorithm flow is shown in Figure 2.

#### 3.1.1. Action Selection Strategy

In order to solve the problem that the agent may choose to execute random actions caused by the constant or decreasing parameter *ε* of a typical action selection strategy in the later stage, thus greatly reducing the convergence speed of the algorithm, an optimized action selection strategy is needed, and the formula is as follows:

(7) $$\begin{array}{c} \pi^{i}\left(s_{t}^{i}\right)=\left\{\begin{array}{cc} a_{\text{random}}, & \text{rand}<\varepsilon ,\\ \underset{a^{\prime }}{\max}Q_{t}^{i}\left(s_{t}^{i},a^{\prime }\right)\text{,} & \text{rand}\geq \varepsilon , \end{array}\right)\\ \varepsilon =\frac{1}{\lambda \bar{t}/\bar{T}}, \end{array}$$

where *π*^*i*^(*s*_*t*_^*i*^) is the best action strategy of the agent belonging to the *i*-th in-state *s*_*t*_ when the *t*-th iterative update is carried out, *a*_random_ is the random selection action, *rand* is the random number with a value range of [0, 1], *λ* is the control rate of *ε* descent, $\bar{t}$ is the current number of training rounds, and $\bar{T}$ is the total number of training rounds.

The article "Research on Intelligent Scheduling Scheme of Aerobics Competition for Multi-Intelligent Decision-Making" was published in 2022. Journal: Comput Intell Neurosci.

#### 3.1.2. Competitive DQN

In deep reinforcement learning, DQN is undoubtedly the most frequently used method, but it is only applicable to a single agent. Facing multiagent, it is obvious that the efficiency of ordinary DQN cannot keep up with a large number of state and action combinations of each agent. Therefore, for multi-intelligent systems, it is necessary to apply competitive DQN as the basic structure to improve the original structure and improve the algorithm efficiency.

Competitive DQN solves the problem that a certain state is immune to any action, which can not affect the subsequent state. It breaks the value combination of state and action, which can improve efficiency. The competitive DQN structure is shown in Figure 3.

Among them, the state value function will have a value equal to 0, and the action advantage function will also have a value equal to *Q*. In order to avoid this kind of situation, it is necessary to reduce the *Q* value, but the order of the action dominance function cannot be changed, so as to reach the degree of freedom without redundancy. The formula is as follows:

(8) $$\begin{array}{c} Q\left(s_{t},a_{t};\theta ,\theta_{V},\theta_{A}\right)=V\left(s_{t};\theta ,\theta_{V}\right)+\left[A\left(s_{t},a_{t};\theta ,\theta_{A}\right)-\frac{1}{N_{A}}\sum_{a^{\prime }}A\left(s_{t},a^{\prime };\theta ,\theta_{A}\right)\right., \end{array}$$

where *Q*(*s*_*t*_, *a*_*t*_; *θ*, *θ*_*V*_, *θ*_*A*_) is the agent in state *s*_*t*_ that executes the *Q* value of action *a*_*t*_ at the *t*-th iterative update. *V*(*s*_*t*_; *θ*, *θ*_*V*_) is the state value function, that is, the value of the state itself, *A*(*s*_*t*_, *a*_*t*_; *θ*, *θ*_*A*_) is the action dominance function, that is, the extra value generated after the corresponding action is selected, and *N*_*A*_ is the number of actions that are likely to occur.

#### 3.1.3. Priority Experience Is Put Back

In the ordinary MFDRL-CTDE algorithm, random sampling is adopted for the step of putting back experience, which undoubtedly subtracts the playback efficiency. Therefore, in order to improve the efficiency of using samples and enhance the function of experience playback, it is necessary to introduce priority experience playback, which can make the samples in the shared experience pool get priority rights, and the possibility of being sampled can be determined. At the same time, high-priority samples are selected many times, which leads to multiple playbacks, which will reduce the diversity of samples. At this time, important sampling weights are needed to solve this problem.

The article "Research on Intelligent Scheduling Scheme of Aerobics Competition for Multi-Intelligent Decision-Making" was published in 2022. Journal: Comput Intell Neurosci.

The formula for judging priority is as follows:

(9) $$\begin{array}{c} \delta_{t}^{ij}=r_{t}^{ij}+\gamma \max Q^{i}\left(s_{t+1}^{i},a^{\prime };\theta_{\text{tar}},\theta_{\text{Vtar}},\theta_{\text{Atar}}\right)-Q^{i}\left(s_{t}^{i},a_{t}^{i};\theta_{\text{val}}^{i},\theta_{\text{Vval}}^{i},\theta_{\text{Aval}}^{i}\right). \end{array}$$

Among them, when *δ*_*t*_^*ij*^ is much greater than 0, it shows that the prediction accuracy has more room for improvement, which makes the convergence efficiency of the algorithm higher. *δ*_*t*_^*ij*^ is time series difference error from the *j*-th sample of the *i*-th agent in the *t*-th iterative update, *r*_*t*_^*ij*^ is an immediate reward from the *j*-th sample of the *i*-th agent in the *t*-th iterative update, *Q*^*i*^(*s*_*t*+1_^*i*^, *a*′; *θ*_tar_, *θ*_Vtar_, *θ*_Atar_) is the Q value obtained by the centralized target of the *i*-th agent, and *Q*^*i*^(*s*_*t*_^*i*^, *a*_*t*_^*i*^; *θ*_val_^*i*^, *θ*_*V*val_^*i*^, *θ*_Aval_^*i*^) is the Q value obtained from the estimation of the *i*-th agent.

The formula for calculating the probability *G*_*ij*_ that a sample is sampled is as follows:

(10) $$\begin{array}{c} G_{ij}=\frac{g_{ij}}{\sum_{k=1}^{N_{g}}g_{ik}}, \end{array}$$

where *N*_*g*_ is the empirical pool capacity.

The formula for calculating sample priority *g*_*ij*_ is as follows:

(11) $$\begin{array}{c} g_{ij}={\left(\left|\delta_{t}^{ij}\right|+\sigma \right)}^{\alpha }, \end{array}$$

where *σ* is a smaller positive number, *α* is degree coefficient, which controls priority and has a value range of [0, 1], and when the value of degree coefficient is 1, it means that sampling is not based on priority, but on random sampling.

The formula of importance sampling weight *w*_*ij*_ is as follows:

(12) $$\begin{array}{c} w_{ij}={\left(N_{g}G_{ij}\right)}^{-\beta }, \end{array}$$

where *β* is the correction degree parameter.

The formula of parameter training target value *y*_*ij*_ is as follows:

(13) $$\begin{array}{c} y_{ij}=\left\{\begin{array}{cc} r_{t}^{ij}, & \text{End of current training round,}\\ r_{t}^{ij}+\gamma \underset{a^{\prime }}{\max}Q^{i}\left(s_{t+1}^{i},a^{\prime };\theta_{\text{tar}},\theta_{\text{Vtar}},\theta_{\text{Atar}}\right), & \text{Others}. \end{array}\right) \end{array}$$

The formula of the corrected loss function is as follows:

(14) $$\begin{array}{c} L\left(\theta_{\text{val}}^{i},\theta_{\text{Vval}}^{i},\theta_{\text{Aval}}^{i}\right)=\sum_{j}w_{ij}{\left[y_{ij}-Q^{i}\left(s_{t}^{i},a_{t}^{i};\theta_{\text{val}}^{i},\theta_{\text{Vval}}^{i},\theta_{\text{Aval}}^{i}\right)\right]}^{2}. \end{array}$$

The article "Research on Intelligent Scheduling Scheme of Aerobics Competition for Multi-Intelligent Decision-Making" was published in 2022. Journal: Comput Intell Neurosci.

## 4. Simulation Experiment

### 4.1. Algorithm Testing

Six typical test functions are selected to calculate and compare the convergence rates of the three algorithms mentioned above. The first three are single-mode benchmark test functions, and the latter three are multimode benchmark test functions. The formula for the test function is as follows:

(15) $$\begin{array}{c} f_{1}\left(x\right)=\sum_{i=1}^{D}x_{i}^{2}-100\leq x_{i}\leq 100,\\ f_{2}\left(x\right)={\sum_{i=1}^{D}\left(\left|x_{i}+0.5\right|\right)}^{2}-100\leq x_{i}\leq 100,\\ f_{3}\left(x\right)=\sum_{i=1}^{D}\left|x_{i}\right|+\prod_{i=1}^{D}\left|x_{i}\right|-10\leq x_{i}\leq 10,\\ f_{4}\left(x\right)=\sum_{i=1}^{D}\left(x_{i}^{2}-10\;\cos\left(2\pi x_{i}\right)+10\right)-5.12\leq x_{i}\leq 5.12,\\ f_{5}\left(x\right)=\frac{1}{400}\sum_{i=1}^{D}x_{i}^{2}-\prod_{i=1}^{D}\cos\left(\frac{x_{i}}{\sqrt{i}}\right)+1-300\leq x_{i}\leq 300,\\ f_{6}\left(x\right)=-20\;\exp\left(-0.2\sqrt{\frac{1}{D}\sum_{i=1}^{D}x_{i}}\right)-\left(\frac{1}{D}\sum_{i=1}^{D}\cos\left(2\pi x_{i}\right)\right)+20+e-32\leq x_{i}\leq 32. \end{array}$$

The average and standard deviation of the three algorithms are calculated after 1000 iterations according to the target test function. The significance of the calculation is that it can reflect the convergence speed of the algorithms and show whether the algorithms are stable or not. The calculation results are shown in Table 1.

The graph of function 1 is shown in Figure 4.

The graph of function 2 is shown in Figure 5.

The graph of function 3 is shown in Figure 6.

The graph of function 4 is shown in Figure 7.

The graph of function 5 is shown in Figure 8.

The graph of function 6 is shown in Figure 9.

It can be seen from the above comparison diagram that the stability and convergence speed of the three algorithms are very close in a single modal function. But, in the multimodal function, it is obvious that Markov does not show good stability, and the convergence rate is very slow. Compared with the improved MFDRL-CTDE algorithm and the common MFDRL-CTDE algorithm, the convergence speed of the former is slightly better than that of the latter, but, for the best performance position, the latter is obviously better than the former, and the latter is more stable. Therefore, in general, the improved MFDRL-CTDE algorithm is superior to the original algorithm.

The article "Research on Intelligent Scheduling Scheme of Aerobics Competition for Multi-Intelligent Decision-Making" was published in 2022. Journal: Comput Intell Neurosci.

### 4.2. Simulation Experiment

#### 4.2.1. Objective Function

Set its standard aerobics action as action sequence *P*, set each person's aerobics action as a series of action sequence *Q*, compare them, and calculate the similarity value.

The formula of similarity evaluation is as follows:

(16) $$\begin{array}{c} \text{DIST}\left(P,Q\right)=\frac{\sum_{r=1}^{R}\text{dist}\left(K_{p_{r}},K_{q_{r^{\prime }}}\right)}{R},\\ \text{Similarity}\left(P,Q\right)=\frac{1}{\text{DIST}\left(P,Q\right)+1}, \end{array}$$

where *R* is the total number of key actions, *K*_*p*_*r*__ is the key action set in standard action sequence *P*, and *K*_*q*_*r*′__ is the key action set in standard action sequence *Q*.

#### 4.2.2. Simulation Experiment and Result Analysis

In the aerobics competition, the movement of each member of the team is set into an action sequence, and the corresponding standard action sequence is compared with it. Suppose there are two aerobics teams participating in the five-person competition and the ten-person competition, respectively. The standard action sequence of aerobics displayed by each team is known. Under the same competition venue, each team completes the display action within 90 seconds at the same time, taking every 10 seconds as a judgment decision point, recording, and setting it into an action sequence to compare its similarity judgment decision.

By taking aerobics as an example, important actions are intercepted as one of the action sequences, and the picture of the intercepted actions is shown in Figure 10.

Put four intercepting actions into the action sequence, which are *a*_*t*_^1^, *a*_*t*_^2^, *a*_*t*_^3^, *a*_*t*_^4^⋯ , and compare the action sequences to calculate the similarity.

Set the volume of the shared experience pool to 2000, the number of playback samples to 10, $\bar{T}=90$, *γ*=0, *α*=0.6, *β*=0.4, *λ*=40.

The similarity comparison data of the five-person group is shown in Table 2.

The similarity comparison data of the ten-person group is shown in Table 3.

The five-person action sequence decision prediction pair is shown in Figure 11.

Therefore, for aerobics competition, the results of the three algorithms for the evaluation scheme decision of the competition action sequence are obvious. With the increase of decision objects, the accuracy of Markov's algorithm is obviously reduced, which coincides with Markov's suitability for a single intelligent decision system. By comparing the MFDRL-CTDE algorithm and the improved MFDRL-CTDE algorithm, it can be clearly seen from the above figure that the improved MFDRL-CTDE algorithm is more stable for the accuracy of predicted values. Although there are very few cases where MFDRL-CTDE predicted values are more accurate than the improved algorithm, most predicted values are still not accurate and stable enough. Therefore, it can be concluded that the improved MFDRL-CTDE algorithm is more stable and efficient for multi-intelligent decision-making systems. In the multi-intelligent decision-making, the system can make good use of all kinds of dance competition action contrast similarity, so that sports competition has a deeper step of development.

The article "Research on Intelligent Scheduling Scheme of Aerobics Competition for Multi-Intelligent Decision-Making" was published in 2022. Journal: Comput Intell Neurosci.

## 5. Conclusion

Compared with MFDRL-CTDE, the improved MFDRL-CTDE algorithm is more suitable for multi-intelligent decision-making. Even after many iterations, the decision-making of the algorithm will not fall into an agent and then execute actions. Obviously, the actions are still executed according to priority, which ensures the efficiency of the algorithm. Markov is more suitable for single intelligent decision-making and cannot be effectively implemented for multi-intelligent decision-making. Therefore, for the scheme scheduling of aerobics competition, the improved MFDRL-CTDE has obvious advantages.

## Figures and Tables

**Figure 1:** Classification diagram of intelligent decision.

**Figure 2:** Flow chart of MFDRL-CTDE algorithm.

**Figure 3:** Competitive DQN structure diagram.

**Figure 4:** Graph of function 1.

**Figure 5:** Graph of function 2.

**Figure 6:** Graph of function 3.

**Figure 7:** Graph of function 4.

**Figure 8:** Graph of function 5.

**Figure 9:** Graph of function 6.

**Figure 10:** Intercept action.

**Figure 11:** Comparison chart of decision prediction of five-person action sequence. The ten-person action sequence decision prediction pair is shown in Figure 12.

**Figure 12:** Comparison chart of decision prediction of ten-person action sequence.

**Table 1:** Test function calculation results table.

Algorithm		*f*_1_	*f*_2_	*f*_3_	*f*_4_	*f*_5_	*f*_6_
Markov	Average	1.17E + 03	1.6832	7.4741	4.80E + 02	0.0357	2.4201
	Standard deviation	1.99E + 03	3.8855	6.2378	2.08E + 02	0.0543	1.2608

MFDRL-CTDE	Average	1.58E + 02	1.6203	8.3282	3.32E + 01	0.0243	2.4001
	Standard deviation	1.70E + 03	3.4943	5.2941	1.8931	0.0083	1.0031

Improved MFDRL-CTDE	Average	1.32E + 02	1.5983	6.2984	3.43E + 01	0.0123	2.1031
	Standard deviation	1.76E + 02	3.0523	5.3823	0.0342	0.0031	0.3134

**Table 2:** Comparison data table of similarity of five-person group.

Time (S)	Actual value (%)	Markov's prediction value (%)	MFDRL-CTDE predictive value (%)	Improved MFDRL-CTDE prediction value (%)
10	80	70	78	80
20	77	68	86	80
30	81	71	75	79
40	85	73	80	83
50	84	69	85	86
60	80	72	75	81
70	79	65	75	79
80	82	70	80	83
90	86	70	81	84

The article "Research on Intelligent Scheduling Scheme of Aerobics Competition for Multi-Intelligent Decision-Making" was published in 2022. Journal: Comput Intell Neurosci.

**Table 3:** Data table of similarity comparison of ten groups.

Time (S)	Actual value (%)	Markov's prediction value (%)	MFDRL-CTDE predictive value (%)	Improved MFDRL-CTDE prediction value (%)
10	75	60	73	71
20	73	61	70	71
30	80	59	85	77
40	78	65	80	80
50	81	68	86	80
60	76	62	70	75
70	80	56	75	81
80	83	60	80	83
90	86	64	80	85

## Data Availability

The experimental data used to support the findings of this study are available from the corresponding author upon request.
